# Association of immune-related adverse events with COVID-19 pneumonia in lung cancer patients receiving immune checkpoint inhibitors: a cross-sectional study in China

**DOI:** 10.1186/s12885-023-11584-w

**Published:** 2023-11-06

**Authors:** Kaijun Che, Chen Hong, Yanqing He, Duanyang Peng, Zhimin Zeng, Anwen Liu

**Affiliations:** 1 Department of Oncology, The Second Affiliated Hospital of Nanchang University, Nanchang, Jiangxi Province PR China; 2 Department of Oncology, The First People’s Hospital of Fuzhou, Fuzhou, Jiangxi Province PR China; 3 Department of Nosocomial Infection Control, The Second Affiliated Hospital of Nanchang University, Nanchang, Jiangxi Province PR China; 4 Jiangxi Key Laboratory of Clinical Translational Cancer Research, Nanchang, Jiangxi Province PR China; 5 Radiation Induced Heart Damage Institute of Nanchang University, Nanchang, Jiangxi Province PR China

**Keywords:** COVID-19 Pneumonia, Immune checkpoint inhibitors, irAEs, Lung Cancer, Omicron variants

## Abstract

**Background:**

Immune checkpoint inhibitors (ICIs) are commonly used to treat lung cancer patients, but their use can lead to immune-related adverse events (irAEs), which pose a challenge for treatment strategies. The impact of irAEs on the incidence of COVID-19 pneumonia in lung cancer patients during the ongoing COVID-19 pandemic is unclear. This study aims to investigate the association between irAEs and COVID-19 pneumonia in lung cancer patients receiving ICIs.

**Methods:**

We conducted a cross-sectional study of lung cancer patients who received ICIs and were infected with COVID-19 due to the Omicron variant between December 2022 and February 2023 in China. We collected data on irAEs and COVID-19 outcomes. Logistic regression analyses were used to calculate odds ratios (ORs) and 95% confidence intervals (CIs) for the association between irAEs and the incidence of COVID-19 pneumonia.

**Results:**

A total of 193 patients were enrolled, with 72 patients (37.30%) in the irAEs group and 121 patients (62.70%) in the non-irAEs group. Twenty-six patients (13.47%) developed COVID-19 pneumonia and 6 patients (3.11%) progressed to severe cases after COVID-19 infection. Multivariate logistic regression showed that the lung cancer patients who experienced irAEs was significantly associated with a higher incidence rate of COVID-19 pneumonia (OR = 9.56, 95%CI: 2.21–41.33; P = 0.0025).

**Conclusion:**

Our study suggests that lung cancer patients receiving ICIs and experiencing irAEs may have a higher risk of developing COVID-19 pneumonia due to the Omicron variant. Therefore, close monitoring of these patients during the COVID-19 pandemic is necessary to mitigate this risk.

## Background

Immune checkpoint inhibitors (ICIs) are commonly used to treat lung cancer, either alone or in combination with chemotherapy and radiotherapy [1, 2]. While ICIs enhance immune function against tumor cells [3, 4], they also carry the risk of immune-related adverse events (irAEs) affecting multiple organs through immunological mechanisms [5]. The incidence of these events varies based on ICI type, dosage, and treatment duration. Immunotherapy-related pneumonitis is a common irAE affecting up to 3%~19% of lung cancer patients treated with ICIs [6–8].

The COVID-19 pandemic has created significant disruptions in healthcare and social and economic systems worldwide [9]. Cancer patients face heightened risks of hospitalization and mortality from the disease due to age-related declines in immune function and immunosuppression from chemotherapy and radiation therapy [10–13]. IrAEs may contribute to these risks by inducing cytokine dysregulation, which can parallel the cytokine storm observed in some cases of COVID-19-induced acute respiratory distress syndrome [14–17]. Previous studies suggest that COVID-19 vaccines are safe for cancer patients receiving anti-PD-1 treatment and that ICIs do not worsen outcomes in cancer patients with COVID-19 [18–22]. Some studies have evaluated the safety and efficacy of ICIs in lung cancer patients with COVID-19 infection [23, 24]. The Omicron variant has presented a new challenge to Chinese healthcare systems and care of cancer patients due to its persistent spread in the end of 2022. However, the impact of irAEs in lung cancer on the incidence of Omicron variant COVID-19 pneumonia remains obscure.

Therefore, this cross-sectional study seeks to investigate the association between irAEs and COVID-19 pneumonia in lung cancer patients infected with the Omicron variant in China. By understanding the impact of irAEs on COVID-19 pneumonia incidence, we can improve the management and monitoring of these patients during the ongoing pandemic.

## Methods

### Design and patients

This cross-sectional study was conducted at the Second Affiliated Hospital of Nanchang University in China between December 8, 2022 and February 1, 2023, during the Omicron variant epidemic. We reviewed lung cancer patients diagnosed with COVID-19, who received at least one cycle of immune checkpoint inhibitors (ICIs), including programmed cell death protein 1 (PD-1)/pro-programmed death-ligand 1 (PD-L1) inhibitors, either as monotherapy or combination therapy at our institution. All enrolled patients had confirmed lung cancer by pathology and COVID-19 diagnosis through reverse transcriptase-polymerase chain reaction (RT-PCR) using nasopharyngeal swabs. Patients diagnosed solely on the basis of rapid antigen testing were excluded. This study adhered to the Declaration of Helsinki principles and followed the Strengthening the Reporting of Observational Studies in Epidemiology (STROBE) reporting guidelines [25]. The institutional ethics committees of the Second Affiliated Hospital of Nanchang University approved the study protocol.

### Data collection

We collected data on patient characteristics, including age, sex, tumor stage, Eastern Cooperative Oncology Group (ECOG) performance status score at the time of COVID-19 infection, previous treatment history, ICI-related data, irAE-related data, and routine blood tests. The Common Terminology Criteria of Adverse Events (version 5.0) was utilized to grade irAE at its peak severity [5]. Solid tumor TNM staging was based on the AJCC staging system’s eighth edition. COVID-19 pneumonia diagnosis was confirmed via chest computed tomography (CT) scans, and patients were categorized based on the NCCN Guidelines for cancer-related infections as having mild, moderate, severe, or critical COVID-19 severity [26].

### Statistical analysis

We used R software (version 3.6.3) to analyze all data. Categorical variables were reported as frequency and percentage, while continuous variables were expressed as mean ± standard deviation. Groups were compared using independent sample t-tests or analysis of variance (ANOVA). Univariate and multivariate logistic regression analyses were conducted to evaluate the connection between immune-related adverse events (irAEs) and COVID-19 pneumonia incidence; Odds ratios (ORs) with 95% confidence intervals (CIs) were reported. Statistical significance was defined as P < 0.05.

## Results

### Patient characteristics

We excluded 46 patients with non-lung cancer, leaving 326 patients diagnosed with both lung cancer and COVID-19 infection for further investigation. Out of these, 133 patients who did not receive immune checkpoint inhibitor (ICI) treatment were excluded, resulting in a total of 193 patients enrolled in the study. Of these, 72 patients (37.30%) experienced immune-related adverse events (irAEs), while 121 patients (62.70%) did not belong to the irAEs group (Fig. 1). Table 1 presents patients’ baseline demographics, clinical, and biochemical characteristics. The median age for the non-irAEs group was 64.55 years, with 85.95% being male. The irAEs group had a median age of 62.83 years, with 86.11% male. Among the entire cohort, 26 patients (13.47%) developed COVID-19 pneumonia, while six (3.11%) progressed to severe cases after COVID-19 infection. We observed a higher incidence rate of COVID-19 pneumonia in the irAEs group compared to the non-irAEs group (27.78% vs. 4.96%, P < 0.01). Furthermore, the irAEs group had a higher incidence rate of different COVID-19 pneumonia grades (P < 0.01).

**Fig. 1:** Flowchart of patient selection. **Abbreviations:** COVID-19, coronavirus disease 2019; ICIs, Immune checkpoint inhibitors; irAEs, Immune-Related Adverse Events

**Table 1:** Baseline characteristics of all enrolled patients

Characteristics	Total Mean (SD)/ Median (Q1-Q3) / N(%)	Without irAEs Mean (SD)/ Median (Q1-Q3) / N(%)	With irAEs Mean (SD)/ Median (Q1-Q3) / N(%)	P
Age (range)year	65.00 (33.00–84.00)	66.00 (60.00–70.00)	64.00 (57.00–69.00)	0.20
**Age year**				0.33
< 70	148 (76.68%)	90 (74.38%)	58 (80.56%)	
≥70	45 (23.32%)	31 (25.62%)	14 (19.44%)	
**Sex**				0.98
Female	27 (13.99%)	17 (14.05%)	10 (13.89%)	
Male	166 (86.01%)	104 (85.95%)	62 (86.11%)	
**Comorbidities**				0.51
No	159 (82.38%)	98 (80.99%)	61 (84.72%)	
Yes	34 (17.62%)	23 (19.01%)	11 (15.28%)	
**ECOG PS**				0.62
≤ 2	183 (94.82%)	114 (94.21%)	69 (95.83%)	
≥ 3	10 (5.18%)	7 (5.79%)	3 (4.17%)	
**TNM stage**				0.28
I-III	43 (22.28%)	30 (24.79%)	13 (18.06%)	
IV	150 (77.72%)	91 (75.21%)	59 (81.94%)	
**Chemotherapy**				0.17
No	24 (12.44%)	12 (9.92%)	12 (16.67%)	
Yes	169 (87.56%)	109 (90.08%)	60 (83.33%)	
**Radiotherapy**				0.18
No	111 (57.51%)	74 (61.16%)	37 (51.39%)	
Yes	82 (42.49%)	47 (38.84%)	35 (48.61%)	
**Targeted therapy**				0.37
No	123 (63.73%)	80 (66.12%)	43 (59.72%)	
Yes	70 (36.27%)	41 (33.88%)	29 (40.28%)	
**Anti-angiogenic therapy**				0.04
No	120 (62.18%)	82 (67.77%)	38 (52.78%)	
Yes	73 (37.82%)	39 (32.23%)	34 (47.22%)	
**COVID-19 pneumonia**				< 0.01
No	167 (86.53%)	115 (95.04%)	52 (72.22%)	
Yes	26 (13.47%)	6 (4.96%)	20 (27.78%)	
**COVID-19 pneumonia grade**				< 0.01
No	167 (86.53%)	115 (95.04%)	52 (72.22%)	
1–2	20 (10.36%)	3 (2.48%)	17 (23.61%)	
3–4	6 (3.11%)	3 (2.48%)	3 (4.17%)	
**WBC (10** ^**9**^ **/L)**	5.66 (4.58–7.13)	5.66 (4.51–7.17)	5.69 (4.71–7.02)	0.95
**Neutrophil(10** ^**9**^ **/L)**	3.67 (2.87–5.03)	3.65 (2.75–4.97)	3.74 (3.13–5.05)	0.68
**Lymphocyte (10** ^**9**^ **/L)**	1.09 (0.81–1.53)	1.13 (0.81–1.50)	1.08 (0.83–1.57)	0.66

**Note**: Comorbidities included chronic obstructive pulmonary disease, hypertension and cardiovascular disease. **Abbreviation**: WBC white blood cell; COVID-19, coronavirus disease 2019; ECOG PS Eastern Cooperative Oncology Group performance status score; irAEs Immune-Related Adverse Events

### Profiles of irAEs

Table 2 showed the types of irAEs in the 72 lung cancer patients. A total of 104 irAE trips were documented after immune checkpoint inhibitor (ICI) treatment. Most common types of irAEs were dermatitis/rash (33.65%), thyroiditis (23.08%), pneumonitis (22.12%), hepatitis (8.65%), colitis (7.69%), and other types (3.85%) in the 72 lung cancer patients. For patients who had multisystem irAEs, the highest grade was considered a priority. Most irAEs were mild, with grade 1 accounting for 50.00% and grade 2 accounting for 29.81%. Eleven patients experienced grade 3 or grade 4 irAEs. No severe (grade 5) irAEs were reported after ICI therapy, with only one patient experiencing grade 1 myocarditis.

**Table 2:** The types of irAEs in lung cancer patients

Types of irAEs	Grade 1	Grade2	Grade 3	Grade 4	Total
Pneumonitis	7	6	4	6	23 (22.12%)
Hepatitis	4	3	1	1	9(8.65%)
Thyroiditis	13	8	3	—	24(23.08%)
Dermatitis/rash	19	11	2	3	35(33.65%)
Colitis	5	2	1	—	8 (7.69%)
Myocarditis	1	—	—	—	1(0. 96%)
others	3	1	—	—	4(3.85%)
**Total**	52(50.00%)	31 (29.80%)	11 (10.58%)	10 (9.62%)	104(100%)

**Abbreviations:** ICI, immune checkpoint inhibitor; irAEs, immune-related adverse events

### Association between irAEs and COVID-19 pneumonia

As shown in Table 3, in the univariate analysis, irAEs (OR = 7.37, 95%CI: 2.80, 19.43; P<0.01) and lymphocyte count (OR = 0.37, 95%CI: 0.15, 0.89; P = 0.03) were associated with a higher incidence of developing COVID-19 pneumonia after infection. However, we did not find a significant association between all-grade irAEs and COVID-19 pneumonia (OR = 1.00, 95%CI: 0.30, 3.29; P = 1.00). In the multivariate analysis, the incidence of COVID-19 pneumonia remained significantly associated with irAEs (OR = 9.56, 95%CI: 2.21,41.33; P = 0.0025) and lymphocyte count (OR = 0.35, 95%CI: 0.14, 0.9; P = 0.0033). Comorbidities (OR = 2.38, 95%CI: 0.76, 7.49; P = 0.14), chemotherapy (OR = 0.64, 95%CI: 0.18, 2.28; P = 0.49), targeted therapy (OR = 2.24, 95%CI: 0.46,10.84; P = 0.32), and anti-angiogenic therapy (OR = 0.73, 95%CI: 0.15, 3.54; P = 0.70) were not significantly associated with COVID-19 pneumonia.

**Table 3:** Univariate and multivariate analyses for risk factors associated with COVID- 19 pneumonia

Variate	COVID- 19 Pneumonia					
	Patients n (%)	Univariate			Multivariate	
		OR (95%CI)	P		OR (95%CI)	P
**Age(years)**			0.98			
< 70	148 (76.68%)	1				
≥ 70	45 (23.32%)	0.98 (0.37, 2.62)				
**Sex**			0.33			
Female	27 (13.99%)	1				
Male	166 (86.01%)	2.11 (0.47,9.50)				
**Comorbidities**			0.06			
No	159 (82.38%)	1			1	
Yes	34 (17.62%)	2.41 (0.95, 6.12)			2.38 (0.76, 7.49)	0.14
**ECOG PS**			0.74			
≤ 2	183 (94.82%)	1				
≥ 3	10 (5.18%)	0.70 (0.09,5.78)				
**TNM stage**			0.69			
I-III	43 (22.28%)	1				
IV	150 (77.72%)	1.24 (0.44, 3.50)				
**irAEs**			< 0.01			
No	121 (62.69%)	1			1	
Yes	72(37.31%)	7.37(2.80,19.43)			9.56 (2.21,41.33)	0.0025
**IrAEs Grade**						
G 0	121 (62.69%)	1			1	
G 1–2	54 (27.98%)	7.37 (2.67, 0.32)	0.0001		0.79 (0.20, 3.11)	0.74
G 3–4	8 (9.33%)	7.37 (1.9,27.54)	0.003		1.0	
**Chemotherapy**			0.09			
No	24(12.44%)	1			1	
Yes	169(87.56%)	0.40 (0.14, 1.13)			0.64 (0.18, 2.28)	0.49
**Radiotherapy**			0.38			
No	111(57.51%)	1				
Yes	82 (42.49%)	0.68 (0.29, 1.62)				
**Targeted therapy**			0.05			
No	123 (63.73%)	1			1	
Yes	70 (36.27%)	2.31 (1.00, 5.33)			2.24 (0.46,10.84)	0.32
**Anti-angiogenic** **therapy**			0.08			
No	120 (62.18%)	1			1	
Yes	73 (37.82%)	2.14 (0.93, 4.92)			0.73 (0.15, 3.54)	0.70
**WBC** **(10** ^**9**^ **/L)**	5.66 (4.58,7.13)	1.08 (0.97, 1.19)	0.16			
**Neutrophil** **(10** ^**9**^ **/L)**	3.67 (2.87,5.03)	1.03 (0.97, 1.09)	0.37			
**Lymphocyte** **(10** ^**9**^ **/L)**	1.09 (0.81,1.53)	0.37 (0.15, 0.89)	0.03		0.35 (0.14, 0.92)	0.033

**Note**: Comorbidities included chronic obstructive pulmonary disease, hypertension and cardiovascular disease. **Abbreviation**: WBC white blood cell; COVID-19, coronavirus disease 2019; ECOG PS Eastern Cooperative Oncology Group performance status score; irAEs Immune-Related Adverse Events; OR Odds ratio; CI, confidence interval; G grade

## Discussion

COVID-19 infection can cause immune dysregulation, leading to excessive inflammation and high levels of pro-inflammatory cytokines [27, 28]. This study examines the impact of Omicron variant COVID-19 on lung cancer patients in China receiving ICIs. Specifically, we conducted a cross-sectional analysis of patients diagnosed between December 2022 and February 2023. Our results confirm that lung cancer patients who develop irAEs while receiving ICIs suffer a higher risk of Omicron variant COVID-19 pneumonia.

There has been growing concern about the potential for unopposed T-cell activation and downstream cytokine excess resulting from the convergence of ICIs treatment toxicity and COVID-19 in cancer patients [28, 29]. In line with this view, our study found that lung cancer patients who developed irAEs while receiving ICIs had a significantly higher incidence of COVID-19 pneumonia compared to those without irAEs (27.78% vs. 4.96%, P < 0.01). It has been suggested that patients who experience irAEs are those who can mount a more robust reconstitution of anticancer immunity [30]. As a result, lung cancer patients receiving ICIs who become infected with COVID-19 may face a higher risk of immune hyperactivation and cytokine storm. Our multivariate analysis revealed that the development of irAEs was significantly associated with a higher incidence rate of COVID-19 pneumonia. Interestingly, previous studies have yielded conflicting results. For example, Mengni Guo et al. reported that COVID-19 infection may pose a risk of severe irAEs in cancer patients receiving ICIs [24]. On the other hand, a registry for thoracic cancers did not find a significant impact of ICIs on COVID-19 outcomes [31, 32]. A New York study reported that prior ICIs therapy was associated with an increased risk of severe respiratory illness and hospitalization among COVID-19 patients [33]. In contrast, a US study of 25 patients found no association between ICIs therapy and COVID-19-related outcomes [20]. Likewise, a prospective study of 44 patients showed that ICIs therapy within 4 weeks of COVID-19 diagnosis trended toward reducing the risk of COVID-19 mortality [34]. Furthermore, a study involving 41 lung cancer patients found no significant association between ICIs therapy and an increased risk of COVID-19 mortality [35]. Differences in cancer types, COVID-19 variants and patient characteristics may account for these discrepancies. However, in our study, we observed a significant difference in the incidence of COVID-19 pneumonia between different grades of irAEs in the univariate analysis. In the multivariate analysis, no difference was observed. This may be attributed to the relatively low number of irAE events, especially in the Grade 3–4 category.

Our study also found that the absolute lymphocyte count was significantly associated with a higher incidence rate of COVID-19 pneumonia (OR = 0.36, 95%CI: 0.14, 0.94; P = 0.04). Prior research has established that reduced CD4+/CD8 + T cells and lymphocyte count are associated with severe COVID-19 [29] and mortality [36]. Meanwhile, the mechanisms leading to irAEs include the expansion of intertumoral and peripheral T-cell receptor repertoire, as well as the mobilization of large numbers of T cells [37]. These findings suggest that there may be an immunological link between irAEs and COVID-19 pneumonia in lung cancer patients, but further mechanistic studies are needed to fully elucidate this relationship.

While our study has limitations - including its retrospective design and small sample size - it provides valuable real-world data from a Chinese institution during a specific timeframe. What’s more, our study specifically focused on lung cancer patients used ICIs. This focus was chosen because distinguishing immunotherapy-related pneumonitis from COVID-19 pneumonia when both occur simultaneously can be challenging, and CT scanning is often necessary for tumor evaluation and monitoring adverse reactions. Our analysis was limited to the Omicron variants (BA.2 and BA.5), and given the emergence of new strains, more investigation is needed to explore the association between irAEs and COVID-19 infection outcomes in cancer patients. Nonetheless, our findings underscore the importance of close monitoring and timely intervention for lung cancer patients receiving ICIs who contract COVID-19.

## Conclusion

In conclusion, our study firstly evaluated the impact of irAEs on COVID-19 pneumonia incidence in lung cancer patients receiving ICI therapy. We found that patients who developed irAEs were at higher risk of contracting Omicron variant COVID-19 pneumonia. This highlights the importance of increased vigilance for COVID-19 infections in this patient population, along with closer monitoring, including timely chest CT scans, and potentially more aggressive treatment if necessary.

## Data Availability

Data are available on request from the corresponding author Zhimin Zeng upon reasonable request (2zm@163.com).

## List of abbreviations

ICIs: immune checkpoint inhibitors
irAEs: Immune-Related Adverse Events
COVID-19: coronavirus disease 2019
PD-1: programmed cell death protein 1 inhibitors
PD-L1: pro-programmed death-ligand 1inhibitors
ECOG: PS Eastern cooperative oncology group performance status score
CT: computer tomography
AJCC: American Joint Committee on Cancer
NCCN: National Comprehensive Cancer Network
OR: Odds ratio
CI: confidence interval
WBC: white blood cell

## References

[1] Gandhi L, Rodriguez-Abreu D, Gadgeel S, Esteban E, Felip E, De Angelis F, Domine M, Clingan P, Hochmair MJ, Powell SF (2018). Pembrolizumab plus Chemotherapy in Metastatic Non-small-cell Lung Cancer. N Engl J Med.

[2] Novello S, Kowalski DM, Luft A, Gumus M, Vicente D, Mazieres J, Rodriguez-Cid J, Tafreshi A, Cheng Y, Lee KH (2023). Pembrolizumab Plus Chemotherapy in squamous non-small-cell Lung Cancer: 5-Year update of the phase III KEYNOTE-407 study. J Clin Oncology: Official J Am Soc Clin Oncol.

[3] Deng T, Zeng G (2020). Immunotherapy with programmed cell death 1 vs programmed cell death Ligand 1 inhibitors in patients with Cancer. JAMA Oncol.

[4] Bagchi S, Yuan R, Engleman EG. Immune Checkpoint inhibitors for the treatment of Cancer: clinical impact and mechanisms of response and resistance. Annual Rev Pathol Mech Disease 2021, 16(1).10.1146/annurev-pathol-042020-04274133197221

[5] Brahmer JR, Lacchetti C, Schneider BJ, Atkins MB, Thompson JA (2018). Management of Immune-related adverse events in patients treated with Immune checkpoint inhibitor Therapy American Society of Clinical Oncology Clinical Practice Guideline. J Oncol Pract.

[6] Gomatou G, Tzilas V, Kotteas EA, Syrigos K, Bouros D. Immune Checkpoint inhibitor-related pneumonitis. Respiration 2020, 99(11).10.1159/00050994133260191

[7] Suresh K, Voong KR, Shankar B, Forde PM, Ettinger DS, Marrone KA, Kelly RJ, Hann CL, Levy B, Feliciano JL (2018). Pneumonitis in non–small cell Lung Cancer patients receiving Immune Checkpoint Immunotherapy: incidence and risk factors. J Thorac Oncol.

[8] Nishino M, Giobbie-Hurder A, Hatabu H, Ramaiya NH, Hodi FS (2016). Incidence of programmed cell death 1 inhibitor-related pneumonitis in patients with Advanced Cancer: a systematic review and Meta-analysis. Jama Oncol.

[9] Pak A, Adegboye OA, Adekunle AI, Rahman KM, Mcbryde ES, Eisen DP. Economic Consequences of the COVID-19 Outbreak: the Need for Epidemic Preparedness. *FRONTIERS MEDIA SA* 2020(8).10.3389/fpubh.2020.00241PMC727335232574307

[10] Bhalla S, Bakouny Z, Schmidt AL, Labaki C, Doroshow DB. Care disruptions among patients with Lung Cancer: a COVID-19 and Cancer outcomes Study. Lung Cancer 2021(7).10.1016/j.lungcan.2021.07.002PMC828406534461400

[11] Kuderer NM, Choueiri TK, Shah DP. Clinical impact of COVID-19 on patients with cancer (CCC19): a cohort study (vol 395, Pg 1907, 2020). The Lancet 2020(10253):396.10.1016/S0140-6736(20)31187-9PMC725574332473681

[12] Bartleson JM, Radenkovic D, Covarrubias AJ, Furman D, Winer DA, Verdin E. SARS-CoV-2, COVID-19 and the aging immune system. Nat Aging.10.1038/s43587-021-00114-7PMC857056834746804

[13] Thakkar A (2021). Association of clinical factors and recent anticancer therapy with COVID-19 severity among patients with cancer: a report from the COVID-19 and Cancer Consortium. Annals of Oncology: Official Journal of the European Society for Medical Oncology.

[14] Garassino MC, Ribas A. At the crossroads: COVID-19 and Immune-Checkpoint Blockade for Cancer. Cancer Immunol Res 2021(3).10.1158/2326-6066.CIR-21-0008PMC805292933452008

[15] Aaab D, Qiang YA, Yw C, Wen Z. Potential protective role of the anti-PD-1 blockade against SARS-CoV-2 Infection. Biomedicine & Pharmacotherapy; 2021.10.1016/j.biopha.2021.111957PMC831594334339917

[16] Moore JB, June CH. Cytokine release syndrome in severe COVID-19. Science, 368.10.1126/science.abb892532303591

[17] Bonomi L, Ghilardi L, Arnoldi E, Tondini CA, Bettini AC. A Rapid Fatal Evolution of Coronavirus Disease-19 in a patient with Advanced Lung Cancer with a long-time response to Nivolumab - ScienceDirect. J Thorac Oncol 2020, 15(6).10.1016/j.jtho.2020.03.021PMC727055232243919

[18] Mei Q, Hu G, Yang Y, Liu B, Yin J, Li M, Huang Q, Tang X, Boehner A, Bryant A et al. Impact of COVID-19 vaccination on the use of PD-1 inhibitor in treating patients with cancer: a real-world study. J Immunother Cancer 2022, 10(3).10.1136/jitc-2021-004157PMC891537935264438

[19] Hibino M, Uryu K, Takeda T, Kunimatsu Y, Shiotsu S, Uchino J, Hirai S, Yamada T, Okada A, Hasegawa Y (2022). Safety and immunogenicity of mRNA vaccines against severe acute respiratory syndrome coronavirus 2 in patients with Lung cancer receiving immune checkpoint inhibitors: a multicenter observational study in Japan. J Thorac Oncol.

[20] Bui AT, Tyan K, Hurder AG, Rahma OE. Impact of COVID-19 on patients with Cancer receiving Immune Checkpoint inhibitors. J Immunotherapy Precision Oncol 2021.10.36401/JIPO-20-34PMC915325435663537

[21] Immune checkpoint inhibitor therapy and outcomes from SARS-CoV-2 infection in patients with cancer: a joint analysis of OnCovid and ESMO-CoCARE registries. Journal for immunotherapy of cancer. 2022, 10(11).10.1136/jitc-2022-005732PMC971641336450384

[22] Widman AJ, Cohen B, Park V, McClure T, Wolchok J, Kamboj M (2022). Immune-related adverse events among COVID-19–Vaccinated patients with Cancer receiving Immune Checkpoint Blockade. J Natl Compr Canc Netw.

[23] Ksienski D, Gupta S, Truong PT, Bone J, Chan A, Alex D, Hart J, Pollock P, Patterson T, Clarkson M. Safety and efficacy of pembrolizumab for advanced nonsmall cell Lung cancer: before and during the COVID-19 pandemic. J Cancer Res Clin Oncol 2022.10.1007/s00432-022-04181-0PMC928135835834010

[24] Guo M, Liu J, Miao R, Ahmed Z, Yu J, Guan J, Ahmad S, Zhou S, Grove A, Manoucheri M (2022). A single Center Retrospective Study of the impact of COVID-19 Infection on Immune-related adverse events in Cancer patients receiving Immune Checkpoint inhibitors. J Immunother.

[25] Vandenbroucke JP, Elm EV, Altman DG, Gøtzsche P, Mulrow CD (2008). The strengthening the reporting of Observational studies in Epidemiology (STROBE) Statement: guidelines for reporting observational studies. BMJ.

[26] .

[27] Postow MA, Sidlow R, Hellmann MD (2018). Immune-related adverse events Associated with Immune Checkpoint Blockade. N Engl J Med.

[28] Bersanelli M. Controversies about COVID-19 and anticancer treatment with immune checkpoint inhibitors. Immunotherapy.10.2217/imt-2020-0067PMC711759632212881

[29] Xu Z, Shi L, Wang Y, Zhang J, Huang L, Zhang C, Liu S, Zhao P, Liu H, Zhu L (2020). Pathological findings of COVID-19 associated with acute respiratory distress syndrome. The Lancet Respiratory Medicine.

[30] Cortellini A, Buti S, Agostinelli V, Bersanelli M. A systematic review on the emerging association between the occurrence of immune-related adverse events and clinical outcomes with checkpoint inhibitors in advanced cancer patients. Semin Oncol 2019(4/5):46.10.1053/j.seminoncol.2019.10.00331727344

[31] Horn L, Whisenant JG, Torri V, Huang LC, Garassino MC (2020). Thoracic cancers International COVID-19 collaboration (TERAVOLT): impact of type of cancer therapy and COVID therapy on survival. J Clin Oncol.

[32] Garassino MC, Whisenant JG, Huang LC, Trama A, Horn L. COVID-19 in patients with thoracic malignancies (TERAVOLT): first results of an international, registry-based, cohort study. The Lancet Oncology; 2020.10.1016/S1470-2045(20)30314-4PMC729261032539942

[33] Robilotti EV, Babady NE, Mead PA, Rolling T, Perez-Johnston R, Bernardes M, Bogler Y, Caldararo M, Figueroa CJ, Glickman MS (2020). Determinants of COVID-19 Disease severity in patients with cancer. Nat Med.

[34] Lee L, Cazier JB, Starkey T, Turnbull CD, Middleton G (2020). COVID-19 mortality in patients with cancer on chemotherapy or other anticancer treatments: a prospective cohort study. The Lancet.

[35] Luo J, Rizvi H, Egger JV, Preeshagul IR, Hellmann MD (2020). Impact of PD-1 blockade on severity of COVID-19 in patients with Lung Cancers. Cancer Discov.

[36] Huang W, Berube J, Mcnamara M, Saksena S, Hartman M, Arshad T, Bornheimer SJ, O’Gorman M (2020). Lymphocyte subset counts in COVID-19 patients: a Meta-analysis. Cytometry Part A: The Journal of the International Society for Analytical Cytology.

[37] Lozano AX, Chaudhuri AA, Nene A, Bacchiocchi A, Earland N, Vesely MD, Usmani A, Turner BE, Steen CB, Luca BA (2022). T cell characteristics associated with toxicity to immune checkpoint blockade in patients with Melanoma. Nat Med.

